This article has been retracted.

# Analysis of Factors Related to Spiritual Psychology and Quality of Life in Patients with Inflammatory Bowel Disease Based on Artificial Intelligence IBD Nursing Technology

**DOI:** 10.1155/2022/7702432

**Published:** 2022-04-11

**Authors:** Shizhen Bao, Wenjia Liu, Li liu, Guifen Jiang, Huan Chen

**Affiliations:** Changzhou Second People's Hospital Affiliated to Nanjing Medical University Gastroenterology, Changzhou 213000, Jiangsu, China

## Abstract

To investigate the characteristics of psychological symptoms in inflammatory bowel disease (IBD), to study the relationship between psychological symptoms and quality of life, and to provide some theoretical basis for the corresponding psychological treatment of IBD patients with psychiatric abnormalities. With the development of artificial intelligence (AI) and its gradual application to the medical field, it has brought new ideas to the medical development, and its research and application in IBD, including ulcerative colitis (UC) and Crohn's disease (CD), is increasing. Machine learning is used to select reasonable models and methods to help the prediction, diagnosis, treatment, and prognosis of IBD. In this study, we improved on the classical unidirectional LSTM model by adding backward and forward LSTM layers, designed a bidirectional LSTM model to improve the shortcomings of unidirectional LSTM with insufficient dependence on the posterior, introduced the contribution rate *α* to adjust the weight matrix of the forward LSTM layer and the backward LSTM layer, and experimentally verified the correctness and superiority of the proposed model. A total of 159 patients with IBD and 89 healthy people were collected and psychologically assessed using the general status questionnaire, the 90-item symptom checklist (SCL-90). Patients with IBD are prone to a combination of obsessive-compulsive, interpersonal, depressive, hostile, and other abnormal psychological symptoms, and their quality of life is significantly reduced; quality of life is mainly affected by disease condition, depression, interpersonal sensitivity, and paranoia, and patients in the active stage of the disease with heavy symptoms of depression, paranoia, and interpersonal sensitivity have low quality of life.

## 1. Introduction

IBD is a nonspecific chronic inflammatory disease of the intestine whose etiology is not well understood, including ulcerative colitis (UC) and Crohn's disease (CD). The number of consultations in China has been increasing rapidly in the last 20 years or so [1, 2]. UC most often occurs in young adults, with a peak incidence of 20–49 years old and little difference between males and females according to Chinese statistics [3], while CD most often occurs in young adults, with a peak incidence of 18–35 years old and slightly more males than females [4], with approximately equal incidence of UC and CD [5]. The clinical manifestations of both diseases are very similar, such as mucopurulent stools, abdominal pain, and various degrees of systemic symptoms, and the diagnosis is made based on a comprehensive analysis combining clinical manifestations, laboratory tests, endoscopy, imaging, and histopathological examinations to exclude infectious and other noninfectious colitis [6].

AI is a branch of computer science that allows computers to perform activities that are normally possible with intelligent beings. AI in a broad sense covers machine learning and robotics [7]. Machine learning (ML) is the development of an algorithm that allows a computer to learn from big data to make predictions about unknown events [8]. Along with the rise of AI, the combination of medical imaging and AI is considered to be the most promising area [9, 10]. Especially in the pathology community, AI is considered to have started a new generation of industrial revolution with faster and more accurate diagnosis, saving medical costs and allowing physicians to devote more time to the analysis of difficult cases [11].

Due to the current difficulties in the diagnosis and treatment of IBD, AI can be well applied to IBD based on big data. This study briefly reviews the current application and progress of AI in IBD, aiming to arouse readers' interest in the research of AI application in IBD.

## 2. Related Work

As a major form of AI, ML is an application that performs iterative modeling by employing several methods [12, 13].

For classification, the most common approach is to use a subset of genes to obtain phenotypic features of interest [14]. In [15], a new and generalization individualized pathway-based classification method, probabilistic pathway score (PROPS) was proposed, which uses a Gaussian Bayesian network to create personalized features reflecting pathway activity and applies these pathway-based features to distinguish between chronic disease and ulcerative colitis, and this method is excellent. The results show that PROPS outperforms existing IBD classifiers and alternative approaches in terms of performance and is useful for distinguishing between UC and CD even when the pathways known to be shared by both show different activities [16]. Resulting in a segmentation method that combines SSL and AI to give a segmentation method that optimally, this method has fewer samples and less training effort than the FSL method, and the segmentation accuracy is higher. Recently, a newly developed feature selection algorithm (doubly randomized preference trial, DRPT) combined with the SVM classifier generated a model to distinguish healthy subjects from UC subjects based on the expression values of 32 genes in colon samples; the model perfectly detected all active cases and showed good performance in the final model for detecting UC performance [17].

## 3. Bidirectional LSTM Neural Network Model

The most widely used character labeling method in academia is the four-word bit labeling set, B, M, E, S, where B (begin) represents the beginning character of the labeled word, *M* (middle) represents the middle character of the labeled word, *E* (end) represents the ending character of the labeled word, and S (single) represents the labeled word as a single character. Determine the corresponding label for each character in the character sequence. A simple model of IBD based on a bidirectional LSTM neural network is shown in Figure 1.

### 3.1. Text Vectorization Layer

To use neural network models to process data, the input data need to be factorized first. There are two main ways of text factorization. The similarity between words cannot be well characterized, which is also known as the lexical gap problem. Word2Vec [18] is a toolkit for acquiring word vectors, which was open-sourced by Google in 2013 and is simple, efficient, and easy to use. The experimental part of this study uses Word2Vec as the first layer to preprocess the input data into word embedding vectors. The word annotation-based word separation method is then based on a local sliding window, assuming that the label of a world greatly depends on the word in its neighboring position.

### 3.2. Bidirectional LSTM Neural Network Layers

The bidirectional LSTM neural network layer consists of two parts: a single-layer LSTM from front to back and a single-layer LSTM from back to front.

Let the window size be *k* and the word vector dimension bed. The text data in the window are fed into a separate LSTM unit by using a trained word embedding lookup table to obtain a distributed representation vector, and this distributed representation vector is fed into a separate LSTM unit from front to back and fed into a separate LSTM unit after inverting the order from back to front. We also introduce a contribution rate variable *α* to adjust the contribution of the two independent one-way LSTM layers to the subsequent data, which is weighted and input to the hidden layer for linear transformation to obtain a vector of equal dimensionality to the label set.

### 3.3. Tag Score Calculation

The IBD problem can be converted into a label classification problem for characters in a character sequence. For each character in a character sequence, the IBD model based on a bidirectional LSTM neural network gives a score for each class of labels it is in.

By common sense, we determine that for the word separation task, the amount of information from the anterior text is not equivalent to the amount of information from the posterior text. *g*_*f*_(*x*^(*t*)^) the former is greater than the latter, that is, the contribution obtained through the anterior to posterior LSTM layer *g*_*b*_(*x*^(*t*)^) is different from that obtained through the posterior to anterior LSTM layer. Therefore, we introduce a contribution rate variable *α* and *α* ≥ 0.5. Under the condition of introducing *α*, the bidirectional LSTM neural network is transformed to obtain an output *y*^(*t*)^, as shown in the following equation.

(1) $$\begin{array}{c} y^{\left(t\right)}=\alpha g_{f}\left(x^{\left(t\right)}\right)+\left(1-\alpha \right)g_{b}\left(x^{\left(t\right)}\right), \end{array}$$

*y*^(*t*)^ then after a linear transformation of the hidden layer, a vector *y*^(*t*)^ equal to the dimensionality of the label set can be obtained to represent *c*^(*t*)^, the scores belonging to each label.

### 3.4. Label Inference Layer

In the {*B*, *m*, *e*, *s*} label system, the distribution of adjacent labels is not independent of each other. For example, the probability of labels B and s after label B is 0, that is, only labels *m* and *E* may appear after label B. Therefore, the method of label transfer weight matrix proposed in [19] is used to represent this dependency, where *A*_*ij*_ represents the weight transferred from label I to label J. The higher the value of *A*_*ij*_, the more likely it is that label I is transferred to label J. Then, if the label sequence of an input character sequence *c*_1:*n*_ in the training dataset is *y*_1:*n*_, the score of the character label sequence is defined as *s*(*c*_1:*n*_, *y*_1:*n*_, *θ*), as shown in the following equation:

(2) $$\begin{array}{c} s\left(c_{1:n},y_{1:n},\theta \right)=\sum_{t=1}^{n}\left(A_{y_{t-1}y_{t}}+{\bar{y}}_{t}\right). \end{array}$$

Let the input sentence be *x*, and the correct tag sequence of the sentence be *y*. Denote the set of all *x* possible tag sequences by *Y*_*x*_. Define the predicted tag sequence with the highest score in *Y*_*x*_ as $\hat{y}$, as shown in the following equation.

(3) $$\begin{array}{c} \hat{y}=\underset{y\in Y_{x}}{\mathrm{argmax}}s\left(x,y,\theta \right). \end{array}$$

### 3.5. Model Training

We define the loss function in terms of $\Delta \left(y_{i},\hat{y}\right)$ as

(4) $$\begin{array}{c} \Delta \left(y_{i},\hat{y}\right)=\sum_{t}^{n}\eta 1\left\{y_{i}^{\left(t\right)}\neq {\hat{y}}^{\left(t\right)}\right\}, \end{array}$$

where $1\left\{y_{i}^{\left(t\right)}\neq {\hat{y}}^{\left(t\right)}\right\}$ indicates when $1\left\{y_{i}^{\left(t\right)}\neq {\hat{y}}^{\left(t\right)}\right\}$ is 1 and 0 otherwise, *η* is the scaling parameter, and $\Delta \left(y_{i},\hat{y}\right)$ indicates the linear correlation of the number of label prediction errors for the input sentence *x*. Let the training set be *T*. We introduce regularization to reduce the degree of overfitting. Let the training set be *T*. We introduce regularization to reduce the degree of overfitting. ‖*θ*‖_2_^2^ is the regularization term of *l*_2_ parametric, which is used to reduce the parameter space and avoid overfitting [20–23]. *λ* is used to control the strength of regularization. The objective function *J*(*θ*) of regularization is

(5) $$\begin{array}{c} J\left(\theta \right)=\frac{1}{T}\sum_{\left(x,y\right)\in t}l_{i}\left(\theta \right)+\frac{\lambda }{2}{\left\|\theta \right\|}_{2}^{2}, \end{array}$$

where

(6) $$\begin{array}{c} l_{\left(\theta \right)}=\max\left(0,s\left(x_{i},{\hat{y}}_{i},\theta \right)+\Delta \left(y_{i},\hat{y}\right)-s\left(x,y,\theta \right)\right). \end{array}$$

Dropout [20] is used during training to control the randomization of some hidden layer nodes in the network from working, while the model is being trained, preventing certain features from being effective only with other specific features.

## 4. Case Study

### 4.1. Information

We randomly collected 159 patients with confirmed IBD in the gastroenterology department of our hospital (IBD group), 102 males and 57 females, aged 16–60 years, including 89 patients with CD, 60 in remission, and 29 in active phase; 70 patients with UC, 33 in remission, and 37 in active phase. In the same period, there were 89 healthy controls, 57 males and 32 females, aged 17–58 years. Inclusion criteria: the IBD group met the diagnostic criteria of the 2012 Guangzhou Consensus on Diagnosis and Treatment of Inflammatory Bowel Disease, aged 16–60 years, and those who could understand and agree to the survey; health control group: the same period of outpatient physical examination center, collected no digestive system, cardiopulmonary system, and other diseases, no mental illness, and no recent major events.

Exclusion criteria: those with combined cardiovascular, cerebrovascular, hepatic, renal, and other systemic diseases that seriously endanger life; those with mental illness; those with infectious, hereditary, metabolic, and endocrine diseases; those with a history of ethanol or drug abuse; pregnant and lactating women; and patients with intestinal tumors. 2 groups were comparable in terms of gender and age [24].

### 4.2. Research Content

The inflammatory bowel disease questionnaire (IBDQ) was developed by Canadian scholars Guyatt et al. It consists of 33 items, including 32 qualitative and semiquantitative questions, measuring intestinal symptoms. The MOSitem short from health survey (SF-36), a total of 36 items, is divided into 8 dimensions, including physical function, physical function, somatic pain, general health, vitality, social function, and emotional function [25].

### 4.3. Results

The IBD group had higher positive rates of SCL-90 factors for mental health somatization, interpersonal relationships, depression, hostility, paranoia, other symptoms, and total score than the control group (*P* < 0.05 to *P* < 0.01). The difference between the two groups was not statistically significant (*P* > 0.05) for obsessive-compulsive, anxiety, fear and psychotic symptoms (Table 1); the IBD group scored higher than the control group for SCL-90 factors somatization, obsessive-compulsive, depression, anxiety, hostility, paranoia, and others (*P* < 0.01). The IBD group had higher SCL-90 scores for all factors in the active phase than in the remission phase (*P* < 0.01) and higher positive rates for somatization, interpersonal sensitivity, depression, anxiety, hostility, and paranoia than in the remission phase (*P* < 0.05 to *P* < 0.01) [26]. Table 1 provides the comparison of SCL-90 factor positivity in the IBD group and control group.

In the SF-36 survey analysis, the IBD group scored lower than the control group in all dimensions except mental health (*P* < 0.01). The total IBDQ score of the enrolled IBD patients is (166.47 ± 29.58), intestinal symptoms (55.18 ± 10.31), general symptoms (23.82 ± 6.144), emotional symptoms (62.54 ± 10.78), and social symptoms (24.92 ± 6.78). Patients with SCL-90 positive IBD had lower scores in total, general, bowel, and affective symptoms compared with those with SCL-90 negative IBD (*P* < 0.01).  Table 2 provides comparison of SF-36 scores between the IBD group and the control group.  Table 3 provides the comparison of IBDQ in SCL-90 positive and negative IBD patients.

A multiple linear regression was performed with quality of life (IBDQ total score) as the dependent variable and education, marital status, gender, age, place of residence, disease condition, whether in school, duration of illness, length of hospitalization, SCL-90 total score, number of positives, somatization, interpersonal sensitivity, depression, anxiety, hostility, paranoia, psychotic, other, obsessive-compulsive, and phobia as independent variables, and the independent variables that entered into the regression equation were disease condition (*b* = –27.163, *P* < 0.01), depression (*b* = –18.583, *P* < 0.01), interpersonal relationship (*b* = 17.653, *P* < 0.01), and paranoia (*b* = –14.316, *P* < 0.01) [27].

## 5. Model Performance and Effect Analysis

In this study, SCL-90 was used to analyze psychological symptoms in patients with IBD, and the results showed statistically significant differences in the positive rates and scores for somatization, interpersonal sensitivity, depression, hostility, paranoia, and others in the IBD group compared to healthy controls. This indicates that people with IBD are more likely to have a combination of abnormal psychological symptoms compared to healthy people. Early on, behavioral changes similar to human mood disorders were found in rats with chronic gastrointestinal inflammation. Later, as more in-depth studies and research on IBD were conducted, it was recognized that psychosomatic factors were closely related to IBD. In an analysis of IBD studies published from 2005 to 2014, 19.1% had anxiety and 21.2% had depression compared to the healthy population and 66.4% had anxiety and 34.7% had depression in active IBD compared to remission [28]. A national survey of a large sample of IBD patients in Canada showed that IBD with generalized anxiety disorder was twice as likely as non-IBD patients.  Figure 2 shows status of different patients.

Patients with IBD are not only prone to a combination of abnormal psychology but also have a variety of components that affect their mental health in many ways. This may be due to the fact that IBD is a chronic disease with recurrent, unpredictable, and systemic disease characteristics, which makes patients suffer from the disease [29]. In addition, although IBD mainly affects the gastrointestinal system, 70% of patients with IBD develop complications such as gastrointestinal perforation or stricture within 10 years of diagnosis, requiring surgical resection or hospitalization [3], incurring high treatment costs, and causing a burden on life [25], which can easily produce symptoms such as anxiety and depression to varying degrees. Patients have a variety of abnormal psychological symptoms, which can be manifested as melancholy and bitterness, loss of enthusiasm for life, reduced activity; increased sense of inferiority, self-blame; hypersensitivity and irritability; and in severe cases, anxiety and suicidal thoughts, as shown in Figure 3.

The results of this study showed that the IBD group was impaired in all dimensions except the mental health dimension compared to normal controls. It indicates that the quality of life of IBD patients is impaired compared to healthy individuals. The IBDQ is a scale developed for IBD patients that better reflects the quality of life of IBD patients in four dimensions, including intestinal symptoms, systemic symptoms, emotional functioning, and social functioning [26]. The results of this study showed that patients with IBD with abnormal psychological symptoms had lower scores in the total score, systemic symptoms, intestinal symptoms, and emotional functioning compared with patients with IBD without abnormal psychological symptoms [30–33]. This suggests that abnormal psychological symptoms can affect patients' systemic and intestinal symptoms and impair their emotional functioning. The reason for this may be that IBD mostly presents with intestinal manifestations such as chronic abdominal pain and diarrhea, blood in stool, and systemic manifestations such as loss of body mass, fatigue, and anemia, which cause patients to become nervous and anxious about the occurrence of related symptoms and thus affect their emotional functioning. Some studies have shown that not only the emotional functioning of IBD patients is affected but also their social functioning is further affected. In the results of the present study, although the differences in social functioning dimensions in the analysis of the IBDQ were not significant, the differences in social functioning dimensions in the analysis of SF-36 were statistically significant [34–37]. The reasons for this may be related to the age differences, small sample size, and relatively concentrated geographical differences in this study, as shown in Figure 4.

The analysis of this study showed that IBDQ of IBD patients was associated with disease activity, depression, interpersonal sensitivity, and paranoia, and in the active phase, depression, interpersonal sensitivity, and paranoia were high, and quality of life was poor. The effects of comorbid psychological factors in IBD patients are extensive not only in terms of quality of life but also in terms of abdominal pain, sleep disturbances, psychotropic medication use, medication nonadherence, and negative disease perception.

## 6. Conclusions

Although AI has achieved brilliant results in many studies, some of them are not very promising. In the construction of AI deep learning models for colonoscopy-assisted diagnosis, the specificity of detecting ulcerative colitis was 67%, which is still lacking. Sometimes, differences are the main confounding bias affecting. Considering the general characteristics of AI models and the unavailability or transparency in computing progress, external validation of AI models is always challenging. Moreover, when an AI model fails in clinical practice, it is also relatively difficult to determine how many errors it will have. Therefore, we should develop predictability of AI models, i.e., the ability to predict the outcome of a model when it performs computational processing.

## Figures and Tables

**Figure 1:** Simple diagram of the bidirectional LSTM neural network model.

**Figure 2:** Status of different patients.

**Figure 3:** Histogram of the distribution of the influence of factors.

**Figure 4:** Quality of life factors for patients with IBD.

**Table 1:** Comparison of SCL-90 factor positivity in the IBD group and control group (*n*, percentage (%)).

Project	IBD (*n* = 159)	Control group (*n* = 89)	*x* ^2^	*P*
Somatization	19	2	6.93	<0.01
Force	65	29	1.67	>0.05
Interpersonal relationship	53	18	4.8	<0.05
Depressed	50	14	7.36	<0.01
Anxious	25	9	1.52	>0.05
Hostile	46	10	10.22	<0.01
Fear	13	2	3.53	>0.05
Paranoid	41	11	6.21	<0.01
Psychotic	19	6	1.71	>0.05
Others	39	10	6.36	<0.05
Total score	48	13	7.47	<0.01

**Table 2:** Comparison of SF-36 scores between the IBD group and the control group ($\bar{x}\pm s$, scores).

Grouping	*n*	Physiological function	Physiological function	Pain	Commonly	Vitality	Sociology	Emotion	Spirit	Total score
IBD group	159	83.08 ± 12.94	43.24 ± 41.12	62.71 ± 23.21	45.24 ± 18.92	43.02 ± 9.2	66.82 ± 22.19	57.23 ± 37.34	60.7 ± 12.59	56.47 ± 10.51
Control group	89	158.906 ± 28.49	21.84 ± 5.77	82.97 ± 15.98	74.33 ± 17.35	47.47 ± 10.95	87.5 ± 14.23	77.15 ± 37.81	60.54 ± 12.68	68.84 ± 8.55
*t*	—	4.74	8.54	6.23	11.96	3.41	7.92	4	0.1	9.48
*P*	—	<0.01	<0.01	<0.01	<0.01	<0.01	<0.01	<0.01	<0.05	<0.01

**Table 3:** Comparison of IBDQ in SCL-90 positive and negative IBD patients ($\bar{x}\pm s$, scores).

Grouping	*n*	Total score	Whole body	Intestine	Emotion	Sociology
SCL-90 negative	63	177.98 ± 27.59	26.84 ± 5.45	57.85 ± 10.26	67.23 ± 9.37	26.04 ± 6.80
SCL-90 positive	96	158.90 ± 28.49	21.84 ± 5.77	53.41 ± 10.06	59.45 ± 10.57	24.18 ± 6.69
*t*	—	4.18	5.45	2.71	4.74	1.7
*P*	—	<0.01	<0.01	<0.01	<0.01	>0.05

## Data Availability

The data used to support the findings of this study are available from the corresponding author upon request.
